# Establishment of Noninvasive Methods for the Detection of *Helicobacter pylori* in Mongolian Gerbils and Application of Main Laboratory Gerbil Populations in China

**DOI:** 10.1155/2022/6036457

**Published:** 2022-03-29

**Authors:** Xiulin Zhang, Cunlong Wang, Yang He, Jin Xing, Yan He, Xueyun Huo, Rui Fu, Xuancheng Lu, Xin Liu, Jianyi Lv, Xiaoyan Du, Zhenwen Chen, Changlong Li

**Affiliations:** ^1^Department of Medical Genetics and Developmental Biology, School of Basic Medical Science, Capital Medical University, Beijing Key Laboratory of Cancer Invasion & Metastasis Research, Beijing, China; ^2^School of Nursing, Dalian Medical University, Dalian, China; ^3^Institute for Laboratory Animal Resources, National Institutes for Food and Drug Control, Beijing, China; ^4^Department of Epidemiology and Biostatistics, School of Public Health, Capital Medical University, Beijing, China; ^5^Laboratory Animal Center, Chinese Center for Disease Control and Prevention, Beijing, China

## Abstract

Identifying *Helicobacter pylori* (*H. pylori*, *Hp*) infection in animals before and after artificial infection influences the subsequent experiment. We established effective and noninvasive detection methods, including the gastric fluid nested polymerase chain reaction (PCR) method and the ^13^C-urea breath test, which can detect *Hp* before modeling *Hp* infection in Mongolian gerbils. We designed a gas collection equipment for gerbils. *Hp* nested PCR was also performed on gastric fluid, gastric mucosa, duodenal contents, and faeces of gerbils challenged with *Hp*. Conventional *Hp* detection methods, including rapid urease assay and immunohistochemistry, were compared. Moreover, we assessed the natural infection of *Hp* in 135 gerbils that had never been exposed to *Hp* artificially from the major laboratory gerbil groups in China. In 10 *Hp* infected gerbils, the positive detection results were 100%, 100%, 90%, and 10% in gastric fluid, gastric mucosa, duodenal contents, and faeces with nested PCR, respectively. A rapid urease test performed on gastric mucosa showed that all animals were infected with *Hp.* Immunohistochemical detection and bacteria culture of gastric mucosa samples that were positive by the nested PCR method also confirmed the presence of *Hp*. 9% (3/35) and 6% (2/31) natural infection rates were found in conventional gerbil groups from the Capital Medical University and Zhejiang Laboratory Animal Center. In conclusion, we established two noninvasive *Hp* detection methods that can be performed before modeling*Hp* infection, including the gastric fluid nested PCR method and the ^13^C-urea breath test.

## 1. Introduction

*Helicobacter pylori* (*H. pylori*, *Hp*) is a gram-negative bacterium that infects more than half of the world's people and is associated with a variety of severe gastric diseases, including gastritis, peptic ulcer, and even adenocarcinoma [1]. Further understanding of the specific mechanism of *H. pylori*-induced gastric cancer is needed.

Researchers have tried to replicate *H. pylori* infection model in animals to study the pathogenesis of *H. pylori* infection in vivo. The colonization efficiency is unsatisfactory in large animals such as monkeys, cats, and dogs [2]. In mice, *H. pylori* infection results in development of gastric adenocarcinoma with some genetically engineered mice or with mice that had been induced with chemical carcinogens in advance [3, 4]. *H. pylori* infection in rats only induces inflammation with preinjury of the gastric mucosa [5]. In 1998, Watanabe and Honda found that Mongolian gerbils can develop gastric adenocarcinoma after long-term *H. pylori* infection without additional chemical carcinogens [6, 7]. Mongolian gerbils are currently recognized as an efficient, cost-effective, and robust rodent model of *H. pylori* infection.

The gerbil model is often used to study the inflammatory response, pathogenic mechanism and therapeutic strategies of *H. pylori* infection. The cancer progression associated with *H. pylori* in gerbils is characterized by erosion, inflammation with neutrophil infiltration, chronic superficial gastritis, atrophic gastritis, intestinal metaplasia, and finally dysplasia and adenocarcinoma, which are similar to those of humans [8, 9]. Nevertheless, in many studies, *H. pylori*-free gerbils were not used or gerbils were not evaluated for natural infection before infection with *H. pylori*. It impacts the reliability and consistency of previous studies [10, 11].

A greater variety of *H. pylori* detection methods have been applied to detect *H. pylori* in human and experimental animals [12]. Bacterial culture was considered the most specific method for the detection of *H. pylori* [12]. However, animals need to be sacrificed first. Immunohistochemistry also requires the animals to be sacrificed. Serum antibody detection and real-time PCR have been widely used clinically [13]. Nested PCR is often performed in gastric mucosa, gastric contents and duodenum to detect *H. pylori* infection, whereas gastric tissue and duodenum can only be obtained after the animals were euthanized. Hence, we developed a gastric fluid nested PCR method that can perform noninvasive *Hp* detection on live gerbils.

^13^C-urea breath test is one of the most reliable noninvasive methods for detecting *H. pylori* infection in humans. *H. pylori* produces urease enzyme and then hydrolyses urea to release CO_2_ and NH_3_. ^13^C-urea breath test can detect the urease production and has been used for the clinical detection of bacteria in antral biopsies [14, 15]. Therefore, we designed a ^13^C-urea breath test equipment for gerbils that are suitable for the size of animals and the volume of expired gas. The ^13^C-urea breath test can detect *Hp* before modelling *Hp* infection in Mongolian gerbils.

In this study, we established two noninvasive *H. pylori* detection methods including the gastric fluid nested PCR method and the ^13^C-urea breath test. We compared these two new methods with conventional *Hp* detection methods and assessed the natural infection of *H. pylori* in gerbils from the major laboratory gerbil groups in China.

## 2. Materials and Methods

### 2.1. Bacterial Strains

*H. pylori* ATCC 43504, *Staphylococcus aureus* ATCC 25923, *Pseudomonas aeruginosa* ATCC 27853, *Escherichia coli* ATCC 25922, *Klebsiella pneumonia* CMCC 46114, *Proteus mirabilis* CMCC 49005, and *Campylobacter jejuni* subsp. ATCC 700819 were provided by the National Institutes for Food and Drug Control. *H. pylori* SS1 was provided by the Capital Medical University. *H. bilis* ATCC51630 was provided by Guangdong Laboratory Animals Monitoring Institute.

### 2.2. Culture of *H. pylori* from the Gastric Mucosa of Mongolian Gerbils

For bacterial culture, the gastric tissue was grounded in Brucella broth (Difco, Detroit, MI, USA) and plated onto Columbia agar (Difco) supplemented with 5% sheep blood and Dent antibiotic supplement (Oxoid, Basingstoke, UK). Incubating the plates at 37°C in a microaerophilic condition for 72 h. Organisms were identified as *H. pylori* by modified Gram staining, oxidase, catalase, and urease reactions and kept frozen at -80°C.

### 2.3. Animals

A total of 69 Mongolian gerbils (6-8 weeks old and 50-60 g) comprising 59 conventional gerbils and 10 specific pathogen-free males were included to establish the *H. pylori* detection methods. The *H. pylori* infection model was replicated in an additional 94 conventional gerbils (6-8 weeks old and 50-60 g). All rodents were from Capital Medical University and fed at a Level II Biosafety laboratory in the Chinese Center for Disease Control and Prevention. Microbiological status of the conventional gerbils and specific pathogen-free gerbils were strictly controlled according to local standards of Beijing. In order to establish *H. pylori-*infected gerbil model, we used 2 × 10^9^ CFU/mL*H. pylori* ATCC 43504 to gavage gerbils for 5 times, 0.5 mL each time. Oral gavage was performed at an interval of 48 h, and the gerbils were fasted for 12 h prior to challenge. The infection method is based on previous reports [6, 9].

In China, the main laboratory gerbils are separately located at the Capital Medical University (CMU), Zhejiang Laboratory Animal Centre (ZJLAC), and Dalian Medical University (DMU) [16, 17]. All colonies originated from Inner Mongolia in China. The screening groups were from CMU (35 conventional gerbils and 23 clean gerbils), ZJCLA (31 conventional gerbils and 26 clean gerbils), and DMU (20 conventional gerbils) [18, 19].

All gerbils are housed in individual ventilated cages (IVC; 461 × 274 × 229 mm; Tecniplast, Milan, Italy) on a 12 h light/dark cycle, with 2 to 3 gerbils in each cage. Females and males were separated and housed separately. The room temperature was maintained at 22~24°C, and the humidity was maintained at 60~70%. The animal experiments were conducted in accordance with the Guidelines of the CMU Animal Experiments and Experimental Animals Management Committee under a protocol approved by the Animal Experiments and Experimental Animal Welfare Committee of CMU (Permit number: AEEI-2016-152).

### 2.4. Sample Extraction and Bacterial Genome

To collect gastric fluid, gerbils were gavaged with 0.5 mL distilled water after fasting for 12 h. A gavage needle was inserted into the stomach, and gastric fluid was extracted into a centrifuge tube within 1 min. The gastric fluid was centrifuged, and the genome was extracted using a microsample genomic DNA extraction kit (Tiangen, Beijing, China). DNA concentration and quality were verified by Nanodrop 2000c (Thermo, USA).

After 10 weeks of infection, the animals were anesthetized with isoflurane (induced with 3%, maintained with 2%, in 30% O_2_/70% N_2_O) and then euthanized. Samples of gastric tissue, gastric contents, duodenal contents, and colonic faeces (0.4 g/each) were collected into 1.5 mL sterile centrifuge tubes, respectively. Genomic DNA was extracted by a microsample genomic DNA extraction kit containing centrifugal adsorption columns (Tiangen, Beijing, China).

Bacterial DNA was extracted using a bacterial genomic DNA extraction kit (Tiangen, Beijing, China).

### 2.5. Nested PCR Primer Design, Amplification, and DNA Sequencing

According to previous reports, we compared different *H. pylori* strains, and the conserved region of *H. pylori* (GenBank ID: NC-000915.1) genome *Urea* gene was selected.

Primers were designed by the primer design software Primer Premier 5. The primers for the first PCR were F1: 5′-AGTAGGGCCATACATAGAAA-3′ and R1: 5′-GACAAAACTCGTAACCGT-3′. Each reaction was performed in a 20 *μ*L reaction volume containing 10 *μ*L Dream Taq Green PCR Master Mix (Thermo Fisher Scientific, Massachusetts, MA), 10 pmol each primer, and 50 ng of the extracted template. The PCR protocol was as follows: 95°C for 5 min, followed by 35 cycles of 95°C for 30 s, 51.3°C for 30 s, and 72°C for 30 s, and a final extension at 72°C for 5 min. The expected PCR product was 499 bp.

The primers for the second PCR were F2: 5′-CATAGTTGTCATCGCTTTT-3′ and R2: 5′-GCGTTGGTTGATAGGC-3′. Each reaction was performed in a 20 *μ*L reaction volume containing 10 *μ*L Dream Taq Green PCR Master Mix (Thermo Fisher Scientific, Massachusetts, MA), 10 pmol of each primer, and 50 ng of the extracted template. The PCR was performed at 95°C for 5 min, followed by 35 cycles of 95°C for 30 s, 51.3°C for 30 s, and 72°C for 30 s, and a final extension at 72°C for 5 min. The expected PCR product was 100 bp.

After matching primers 1 and primers 2 of nested PCR with *Helicobacter* species (taxid: 209) on the GenBank database, we confirmed that the matching sequences only exist in *H. pylori*.

The nested PCR amplification product was electrophoresed in 2% agarose gel (Amresco, USA); Takara 50 bp DNA Ladder was used as a molecular mass marker.

DNA sequencing was completed by Beijing Tianyihuiyuan Life Science & Technology Inc. Alignments were performed between nested PCR production sequences and sequences in GenBank.

*H. pylori* ATCC 43504 with a concentration of 2 × 10^8^ ~ 2 × 10^1^ CFU/mL, *Staphylococcus aureus* ATCC 25923, *Pseudomonas aeruginosa* ATCC 27853, *Escherichia coli* ATCC 25922, *Klebsiella pneumonia* CMCC 46114, *Proteus mirabilis* CMCC 49005, *Campylobacter jejuni* subsp. ATCC 700819, and *H. pylori* SS1 were used as templates for nested PCR according to the above conditions, respectively.

### 2.6. Establishment of the 13C-Urea Breath Test Detection Threshold

Gerbils were challenged with *H. pylori* by oral gavage at concentrations of 2 × 10^9^ CFU/mL, 2 × 10^7^ CFU/mL, 2 × 10^5^ CFU/mL, 2 × 10^3^ CFU/mL, and 2 × 10^1^ CFU/mL and sterile saline. Each concentration treatment group contained three animals. Gerbils were placed immediately into a holder tube. The holder tube was connected to a gas propulsion device and a gas collecting device. The gas exhaled by a gerbil for 10 min was collected as the background gas with a ventilation of 0.5 mL/s. The gerbil was removed and was gavaged with 0.8 mg/mL urease solution (Haidewei, Shenzhen, China), and the gerbil was placed back into the holder tube immediately. Sample gas was collected in the same way. Finally, the ^13^C tester (Haidewei, Shenzhen, China) was inserted into the gas bag, and the delta-over-baseline (DOB) value was measured.

### 2.7. Other *H. pylori* Detection Methods

A rapid urease detection kit (SanQiang, China) was performed on gerbil gastric tissue.

Immunohistochemistry and Warthin-Starry silver staining were also performed with gastric tissue to detect *H. pylori*. The gastric tissue was embedded in paraffin and cut into 4 *μ*m-thick sections. Pyloric gastric sections were immunostained for *H. pylori* with primary antibodies (1 : 30 dilution, Batch B-0471, DAKO, Glostrup, Denmark). The Warthin-Starry silver staining kit was purchased from Solarbio (Beijing, China).

### 2.8. Statistical Analysis

ROC (receiver-operating characteristic) curve analysis was used to determine the cut-off value of the detection threshold of the ^13^C-urea breath test. The sensitivity, accuracy, and specificity of the ^13^C-urea breath test methods and nested PCR were compared with several conventional detection methods. All analyses were performed using Graph Pad Prism 8.

## 3. Results

### 3.1. Sensitivity and Specificity Assay of Nested PCR

The results showed that target fragments could be amplified from *H. pylori* at a concentration of 2 × 10^2^ ~ 10^8^ CFU/mL (Figure 1(a)). The lowest concentration of *H. pylori* that can be detected is 2 × 10^2^ CFU/mL and the total PCR reaction volume is 20 *μ*L, containing 4 CFU of bacteria. The expected band can only be observed in *H. pylori* but not in other bacteria (Figures 1(b) and 1(c)). In order to exclude the influence of other bacteria including *Helicobacter* species, we compared the target fragments amplified by nested PCR. The GenBank database was used to perform BLAST analysis on the sequencing results to confirm that the nested PCR amplified fragments were specific fragments of *H. pylori*. Taken together, nested PCR detection method for *H. pylori* has high sensitivity and specificity.

### 3.2. Detection of *H. pylori* Infection by Nested PCR

After 10 weeks of infection with *H. pylori*, the gastric fluid of 10 pathogen-free gerbils was extracted. Gastric tissue, duodenal content, and faecal samples were collected after euthanizing the gerbils. DNA extraction, PCR amplification, and gel electrophoresis were performed on all the samples.

The expected band of the first PCR amplification was 499 bp, and 30% (3/10) of the gastric fluid samples were positive (Figure 2(a)) The expected band of the second PCR amplification was 100 bp. After agarose gel electrophoresis analysis, 100% (10/10), 100% (10/10), 90% (9/10), and 10% (1/10) of the gastric fluid, gastric tissue, duodenal content, and faecal samples were positive for the 100 bp band (Figures 2(b), 2(c), 2(d) and 2(e)).

### 3.3. Results from the Mongolian Gerbil Screening Groups

In order to investigate the natural infection of *H. pylori* in Chinese laboratory gerbils, we performed nested PCR detection of *H. pylori* in gastric fluid and gastric tissue of the main Chinese laboratory gerbil populations. There were three conventional gerbils infected with *H. pylori* at CMU, while the positive rate was 9% (2/35); two conventional gerbils were infected with *H. pylori* at ZJCLA with a 6% (1/31) positive rate. However, the clean gerbils at CMU and ZJCLA and the conventional gerbils at DMU were not infected with *H. pylori* as determined by evaluation of gastric fluid samples with the nested PCR detection method (Table 1). These observations suggested the presence of natural infection of *H. pylori* among laboratory gerbils in China, although the positive rate was low.

### 3.4. Establishment of the Mongolian Gerbil ^13^C-Urea Breath Test and Detection Threshold

*H. pylori* can produce abundant urease enzymes that hydrolyse urea to release CO_2_ and NH_3_. The hydrolysed urea will form ^13^CO_2_ after taking ^13^C-urea capsules orally and enter the lungs with blood and be discharged by gas. Based on this principle, we designed a ^13^C-urea breath test gas collection device (Figure 3(a)) for gerbils that consists of a gerbil holder tube, a gas propulsion device and a gas collecting device. We can determine whether the gerbils are infected with *H. pylori* by detecting the ^13^C in the exhaled gas before and after taking the ^13^C-urea solution. We then studied the relationship between the DOB value and the dose of ^13^C-urea, *H. pylori* concentration and time. The DOB value increased with increasing doses of ^13^C-urea (Figure 3(b)). With the increase in detection time after gavage, the DOB value reached a peak and then gradually decreased (Figure 3(c)). The DOB value increased with increasing *H. pylori* concentration (Figure 3(d)). By detecting the change in DOB with different amounts of *H. pylori* (Figure 3(e)), we determined that by collecting the exhaled gas of gerbils within 10 min after a gavage of 0.5 mg/mL ^13^C-urea solution, the gerbils were considered to be *H. pylori-*positive if DOB > 7.

### 3.5. Detection of *H. pylori*-Infected Gerbils

We established an *H. pylori*-infected Mongolian gerbil model in which the presence of *H. pylori* was evaluated every 5 weeks after infection for 85 weeks (Table 2). The ^13^C-urea breath test showed that 50% (47/94) of gerbils were infected with *H. pylori*, while the positive rate of detection in the gastric mucosa by nested PCR was 95.2% (89/94). Nested PCR showed a 100% positive rate of *H. pylori* infection after 15 weeks. 47 animals that were considered positive by the ^13^C-urea breath test also tested positive by nested PCR. The detection rate of nested PCR in gastric tissue was higher than that of the ^13^C detection method.

### 3.6. Other *H. pylori* Detection Methods

To verify the accuracy of the nested PCR method, immunohistochemistry and rapid urease test were used for comparison in the present study. The rapid urease test showed that the detection rate of 10 animals infected with *H. pylori* was 100% (Table 3). We observed *H. pylori* in gerbils that were *H. pylori*-positive by nested PCR and the ^13^C-urea breath test at the same time through immunohistochemistry (Figure 4). *H. pylori* was cultured and identified from the gastric mucosa of 5 gerbils that were determined to be *H. pylori*-positive by nested PCR performed on gastric fluid and gastric tissue (Figure 5). Bacterial culture proves the presence of *H. pylori*.

## 4. Discussion

Though the transmission route of *H. pylori* infection remains unclear, it is generally believed that the transmission of *H. pylori* person-to-person mainly occurs via the oral-oral or faecal-oral route [20]. Mongolian gerbils are a good animal model for studying *H. pylori* infection and transmission because of the tumor progression associated with *H. pylori* in gerbils is similar to that of humans [9, 21]. Besides, gerbils are often kept as pets for children who are susceptible to *H. pylori* [22].

In Charles River Laboratories International, Inc. (Wilmington, USA)'s latest Gerbil VAF Report, 100.0% (72/72) of gerbils were positive for *Helicobacter* species through PCR detection. Our general survey of the major Mongolian gerbil population in China also showed the natural infection of *H. pylori* through the gastric fluid nested PCR detection method. The positive rate was highest (9%) in the conventional gerbils at the Capital Medical University. In rodents, direct transmission of *H. pylori* occurs from challenged mice to unchallenged mice via saliva and faeces in a single cage [23]. Studies have found that *H. pylori* infection in Mongolian gerbil pups are transmitted by the faecal-oral route from an infected mother [21]. Mongolian gerbils are susceptible to *H. pylori* as previously reported [6]. We also found that the rate of colonization in the Mongolian gerbils infected with *H. pylori* was 100% after 10 weeks. Furthermore, Mongolian gerbils have been kept as pets for children, and the transmission of *H. pylori* between humans and pets has been reported [24]. It is necessary to determine the prevalence of *H. pylori* in pet gerbils through noninvasive detection methods. In addition to being used in the investigation of *H. pylori*, Mongolian gerbils are also considered to be a good animal model for studying hearing loss and brain ischemia. In these studies, unexpected results may be produced since *H. pylori* infection leads to increased expression of IL12 and IFN*γ* in Mongolian gerbils, which seriously affects the accuracy of experimental results [25–27]. Besides, *H. pylori* infection may induce extragastric diseases, making it difficult to determine the health status of experimental gerbils [28]. Though *H. pylori* detection before replicating the *H. pylori*-infected model in gerbils is necessary, we found few studies that used *H. pylori*-free gerbils or detected the natural infection before challenge with *H. pylori* [10, 11]. However, we cannot confirm whether the animal had been infected after modelling for a long time unless the animal was sacrificed, which affected the efficiency of modelling and did not conform to the “3R principle” (reduce, refine, and replace). Therefore, there is an urgent need for the detection of *H. pylori* infection before modelling through a more accurate and noninvasive detection method and for long-term detection [29].

Hence, we developed a method of gastric fluid nested PCR that only needs to extract the gastric fluid of live gerbils through gavage needle without harming the animals [12]. The positive rate of detection from gastric fluid with nested PCR was consistent with the results of the rapid urease detection method, indicating that the gastric fluid nested PCR method had convincing accuracy.

Chronic *H. pylori* infection can reduce the secretion of gastric acid and allow the growth of the gastric bacterial community [30]. The extracted gastric fluid may contain other bacteria besides *H. pylori*. We amplified several common bacterial DNAs including *H. bilis* with nested PCR primers, and no target fragments were detected [31]. After using GenBank database to match primer 1 and primer 2 of nested PCR to *Helicobacter* species (taxid:209), we found that the matching sequence of both primer 1 and primer 2 only existed in *H. pylori*. Thus, we confirmed that the nested PCR method is specific to *H. pylori*. The gastric fluid nested PCR method has high specificity. Considering the primers are a target to bacteria themselves, nested PCR could theoretically be applied in rodents which needs further investigation.

Nested PCR amplification was then performed with genomes from different concentrations of *H. pylori*. Target fragments could be amplified successfully from *H. pylori* at a concentration of 2 × 10^2^ ~ 2 × 10^8^ CFU/mL, that is, the copies of the bacterial genome are 10^6^~1, indicating that the nested PCR method has a high sensitivity. In Figure 1(a), agarose gel electrophoresis was performed for the second PCR product of nested PCR. Two bands of PCR products were shown, the lower band was the target band of the second PCR, with a size of 100 bp, and the upper band was the unreacted DNA template, with a size of 499 bp from the first PCR.

The positive rate of *H. pylori* infection determined by nested PCR was different in different parts of the alimentary canal. During the gavage process, *H. pylori* entered the junction of the duodenum and stomach with water or food, which caused a high positive rate of detection in the duodenal contents. The positive rate of *H. pylori* in faeces was low which may be due to the PCR inhibitors contained in the faecal material. Bacterial culture was considered the most specific method for the detection of *H. pylori*; therefore, we performed bacterial culture from gastric mucosa of 5 gerbils. Nested PCR of gastric tissue and gastric fluid has determined that all the gerbils are *H. pylori* positive. Gram staining, oxidase, catalase, and urease reactions confirmed the presence of *H. pylori.* These results demonstrate the reliability of the nested PCR method.

^13^C-urea breath test has been applied in clinic and in many experimental animals except for gerbils, such as *H. pylori* infected mice model and barrier born pigs [32, 33]. Although the detection standards are different due to the differences in size of animals and in volume of expired gas, the ^13^C-urea breath test is harmless and reliable in these animals. Hence, we designed a gas collection equipment suitable for gerbils and defined the detection method and threshold of gerbil ^13^C-urea breath test.

In our research, when gerbils were examined every 5 weeks after infection for 85 weeks, the ^13^C-urea breath test showed that 50% of gerbils were infected with *H. pylori*, while the positive rate of gastric mucosa by nested PCR was 95.2%. The accuracy of the ^13^C-urea breath test is unsatisfactory because the urease test basically depends on bacterial density [34]. It is difficult to detect the presence of *H. pylori* by ^13^C-urea breath test at a very low density. Meanwhile, in our study, the air in the holder tube of gerbil gas collection equipment diluted the ^13^CO_2_ concentration. As there is no special ^13^C-urea breath equipment for rodents, we have no choice but to select ^13^CO_2_ detector for humans. We aim to improve the detection method and establish a better detection threshold in the future.

## 5. Conclusions

In conclusion, there is a strong need to detect *H. pylori* with a noninvasive method in gerbils before replicating the model of *H. pylori* infection because of the considerable natural infection rate and acute effects in animal colonies and individuals after infection. It can improve the validity, reliability, and consistency of subsequent experiments and lay the foundation for research on the pathogenic mechanism and a therapeutic strategy for gastric disease caused by *H. pylori*.

## Figures and Tables

**Figure 1:** Sensitivity and specificity assays of nested PCR. (a) The nested PCR electrophoresis map of different concentrations of *H. pylori*. The target band was 100 bp. The concentrations of *H. pylori* in wells 1~8 were 2 × 10^8^ CFU/mL, 2 × 10^7^ CFU/mL, 2 × 10^6^ CFU/mL, 2 × 10^5^ CFU/mL, 2 × 10^4^ CFU/mL, 2 × 10^3^ CFU/mL, 2 × 10^2^ CFU/mL, and 2 × 10^1^ CFU/mL. (b) The nested PCR electrophoresis map of different bacteria. The bacterial samples in wells 1-9 were *H. pylori* ATCC 43504, *H. pylori* SS1, *Staphylococcus aureus* ATCC 25923, *Pseudomonas aeruginosa* ATCC 27853, *Escherichia coli* ATCC 25922, *Klebsiella pneumonia* CMCC 46114, *Proteus mirabilis* CMCC 49005, *Campylobacter jejuni* subsp. ATCC 700819, and nucleotide-free water. (c) The nested PCR electrophoresis map of different bacteria. The bacterial samples in wells 1-3 were nucleotide-free water, *H. pylori* ATCC 43504, and *H. bilis* ATCC51630.

**Figure 2:** The detection of *H. pylori* in Mongolian gerbils by different PCR methods. (a) Electrophoresis of PCR products from gastric fluid samples; (b) electrophoresis of nested PCR products from gastric fluid samples; (c) electrophoresis of nested PCR products from gastric mucosa samples; (d) electrophoresis of nested PCR products from duodenum content samples; and (e) electrophoresis of nested PCR products from colonic stool samples. 1-10 are the numbers of 10 different gerbils.

**Figure 3:** The detection threshold of gastric fluid nested PCR ((b–d) *n* = 3; (c) *n* = 5). (a) Mongolian gerbil gas collection; (b) the relationship between CO_2_ DOB value and ^13^C-urea concentrations; (c) the relationship between CO_2_ DOB value and test time; (d) the relationship between CO_2_ DOB value and *H. pylori* concentrations; and (e) the relationship between different *H. pylori* concentrations in Mongolian gerbils and test time with the ^13^C-urea breath test.

**Figure 4:** Immunohistogram of *H. pylori* in gastric mucosa. (a) Blank control, ×400; (b) negative control, ×400; (c) experimental group, ×400; (d) blank control, ×1000; (e) negative control, ×1000; and (f) experimental group, ×1000. (g) Warthin-Starry silver staining on gastric mucosa of *H. pylori* infected gerbil, ×1000.

**Figure 5:** (a). Electrophoresis of nested PCR products from gastric tissue and gastric fluid samples of 5 *H. pylori*-infected gerbils. 1–5 are the nested PCR products of gastric tissue, 6-10 are the nested PCR products of gastric fluid, respectively. (b) Gram staining of bacteria cultured from *H. pylori*-infected gerbils' gastric mucosa, ×1000. (c–e) Oxidase, catalase, and urease reactions of bacteria cultured from *H. pylori*-infected gerbils' gastric mucosa. 1–5 is the number of gerbils. 6 is the negative control. (c) Oxidase reaction. (d) Catalase reaction. (e) Urease reaction.

**Table 1:** The *H. pylori* infection results in different Mongolian gerbil groups.

Name of group	Capital Medical University conventional animal	Capital Medical University clean animal	Dalian Medical University conventional animal	Zhejiang Provincial Experimental Animal Center conventional animal	Zhejiang Provincial Experimental Animal Center clean animal
Number of positive samples from gastric fluid nested PCR	1	0	0	1	0
Number of positive samples from gastric tissue nested PCR	2	0	0	1	0
Total number	35	23	20	31	26
Infection rate	**9%**	**0%**	**0%**	**6%**	**0%**

**Table 2:** The *H. pylori* infection results in different Mongolian gerbil groups every 5 weeks after infection for 85 weeks.

Week after infection	Total number of samples	Number of positive samples via ^13^C detection methods	Number of positive gastric tissue samples via nested PCR
5	6	2	2
10	6	2	5
15	6	3	6
20	5	0	5
25	6	4	6
30	6	0	6
35	6	6	6
40	5	2	5
45	5	5	5
50	4	3	4
55	5	1	5
60	6	0	6
65	6	4	6
70	6	1	6
75	6	5	6
80	5	5	5
85	5	4	5
Total	94	47	89
%	**100.00%**	**50.00%**	**95.20%**

**Table 3:** Comparison of the results of different methods for the detection of *H. pylori* in Mongolian gerbils.

No.	Gastric fluid PCR	Gastric fluid nested PCR	Gastric mucosa nested PCR	Duodenum content nested PCR	Faeces nested PCR	Rapid urease assay
1	+	+	+	+	+	+
2	+	+	+	+	-	+
3	-	+	+	+	-	+
4	-	+	+	+	-	+
5	-	+	+	+	-	+
6	-	+	+	+	-	+
7	+	+	+	+	-	+
8	-	+	+	+	-	+
9	-	+	+	+	-	+
10	-	+	+	-	-	+
Positive	30%	100%	100%	90%	10%	100%

Notes: “+” means positive; “-” means negative.

## Data Availability

All data, models, and code generated or used during the study appear in the submitted article.
